The article "Computed Tomography-Based Prediction of Lumbar Pedicle Screw Loosening" was published in 2023. Journal: Biomed Res Int.

# Computed Tomography-Based Prediction of Lumbar Pedicle Screw Loosening

**DOI:** 10.1155/2023/8084597

**Published:** 2023-01-25

**Authors:** Li Shu, Xiaoyuan Wang, Lei Li, Abudunaibi Aili, Rui Zhang, Wenge Liu, Aikeremujiang Muheremu

**Affiliations:** ^1^Orthopedic Research Center, Sixth Affiliated Hospital of Xinjiang Medical University, Urumqi, Xinjiang 86830001, China; ^2^Intensive Care Unit, Wuxi Xinrui Hospital (Wuxi Branch of Ruijin Hospital), Wuxi, China; ^3^Department of Orthopedics, Union Hospital of Fujian Medical University, China

## Abstract

**Objective:**

Pedicle screw loosening is one of the main complications after pedicle screw fixation. However, there are few reliable measures for prediction of screw loosening. The current study was carried out to find an effective method to use preoperative CT scanning as a predictor of screw loosening in the elderly patients and provide guidance for preoperative surgical planning.

**Methods:**

Patients who were treated with lumbar pedicle screw fixation procedure in our department for degenerative lumbar disorders between January 2015 and January 2021 were retrospectively included in the current study. CT scan attenuation of each vertebra was measured with Hounsfield units (HU). Screw loosening was determined in postoperatively X-ray tests. One-way analysis of variance (ANOVA) and receiver operating characteristic (ROC) curve analysis were carried out with IBMSPSS 24.00 software.

**Results:**

Screw loosening was observed in 44 of 215 patients (124 male, 91 female, average age 58.4 ± 7.6 years) during a mean follow-up time of 19.0 ± 11.2 months (range 12-32 months). No significant differences were found among the patients concerning patient gender, BMI, habit of smoking, and whether or not the patient had diabetes or suffered from spondylolisthesis (*P* > 0.05). The average HU value of lumbar vertebra was 122.4 ± 32.8 HU in the screw loosening group and 142.4 ± 38.2 HU in the control group, and the difference was significant (*P* < 0.01). ROC curve analysis revealed that the average HU value of L1-L5 has a relatively larger area under the curve (AUC) of 0.689 (95% CI: 0.605-0.773). With the sensitivity of 68% and specificity of 57%, a HU cut-off value of ≤124 HU is a plausible cut-off point to predict screw loosening.

**Conclusions:**

A prospective CT scan HU value-based prediction can be used to decide whether or not to use screw augmentation methods. A cut-off L1-L5 average HU value of 124 HU can be used as an independent risk factor for screw loosening in instrumented lumbar vertebra. More predictive indexes should be involved to achieve higher sensitivity and specificity in future clinical practice.

The article "Computed Tomography-Based Prediction of Lumbar Pedicle Screw Loosening" was published in 2023. Journal: Biomed Res Int.

## 1. Introduction

Treatment of various degenerative spinal diseases such as degenerative scoliosis, lumbar spinal stenosis, and spondylolisthesis involves surgical intervention, and pedicle screw fixation is the current standard technique to achieve adequate stabilization after removing a significant part of the spinal structure [1, 2]. After spinal surgeries involving screw fixation, screw loosening is one of the main complications and the cause of pain, morbidity, and decline of life quality [3–5]. Although augmentation of pedicle screws with bone cement or the application of expandable screws can be used to avoid screw loosening, those measures increase the risk of fatal cement embolism and difficulty in revision surgery [6, 7]. Therefore, it is essential to apply those preventive measures for screw loosening only in patients with high probability of screw loosening.

Previous investigations have demonstrated that patients with osteoporosis are at much higher risk of screw loosening than patients with normal bone mineral density because of the significantly reduced integration of the screws at the screw-bone interface [8–10]. As a diagnostic tool for osteoporosis, computed tomography (CT) Hounsfield unit (HU) values have been used in the evaluation of bone mineral density for several decades. Significant correlation was reported between HU value and DXA-based results of bone mineral density [11]. In our previous research, we found relevance between the incidence of screw loosening and the HU value of sacrum after surgeries involving sacral spinal surgeries [12]. However, there are few reports on the relations between HU value and loosening of lumbar pedicle screws. In the current research, to evaluate the applicability of preoperatively obtained CT scan HU value as a predictor of screw loosening after spinal surgeries, we have retrospectively reviewed patients who received surgical intervention with rigid pedicle screw fixation and found the correlation between HU value of different lumbar vertebrae and the incidence of pedicle screw loosening during a follow-up of up to at least 12 months.

## 2. Materials and Methods

### 2.1. Patient Inclusion and Exclusion

All the procedures were approved by the ethical committee of the Sixth Affiliated Hospital of Xinjiang Medical University, and written consent was achieved from the patients before the treatment. Patients who were treated in our hospital with pedicle screw-based lumbar spine surgeries between January 2015 and January 2021 were retrospectively included in the current study. Other indications for inclusion are as follows: had pre- and postoperative CT scans, followed up for at least 12 months; patients with previous history of spinal surgery, patients with congenital scoliosis, spinal fracture, spine tumor, and ankylosing spondylitis; patients with other conditions that may affect bone metabolism such as long-term steroid application; patients with insufficient screw anchorage; and patients who received revision surgery within a year due to infection, hematoma, neural injury, and adjacent level disk degeneration.

The article "Computed Tomography-Based Prediction of Lumbar Pedicle Screw Loosening" was published in 2023. Journal: Biomed Res Int.

### 2.2. Outcome Assessment

All CT scans were performed in our Hospital's Department of Radiology. All the patients received a CT scan (GE 32 row spiral CT, USA). Voltage of the Scantron was 120 kV. Two independent examiners used PACS system (GE, USA) to measure the HU value. Besides radiological parameters, basic patient demographic data including patient age, height, and weight were recorded, and the body mass index (BMI) was calculated.

A region of interest (ROI) within the cortex of vertebra was determined on a horizontal plane of at the level of pedicle, from which attenuation in HU was computationally generated (Figure 1).

All the patients received X-ray scans during and at the end of follow-up visits. Two senior spine surgeons independently evaluated screw loosening and bone fusion. More than 1 mm of clear zone around screw was used as a reference to diagnose screw loosening. Nonfusion was diagnosed when anterior translation was greater than 3 mm, rotation more than 5°, or there was no continued trabecular bone in sagittal flexion-extension X-ray film.

### 2.3. Statistical Analysis

Statistical calculations were performed using SPSS 24.0 (IBM SPSS Corporation, Chicago, Illinois). Intraclass correlation coefficient (ICC) was used to test if the measured HU values are similar between the two independent researchers. Normal distribution was reviewed prior to statistical analyses. Continuous variables were recorded as mean ± standard deviation. Quantitative measures were recorded as percentage. One-way ANOVA was applied to compare the variables between groups. Quantitative data was analyzed by *X*^2^ and Fisher's exact test. ROC curve analysis was carried out to evaluate the diagnostic value of CT scans.

## 3. Results

A total of 215 (124 male, 91 female, average age 58.4 ± 7.6 years) patients were included in the final analysis. Indication for surgery includes spondylolisthesis, spondylodiscitis, degenerative scoliosis, or spinal stenosis. The mean duration of the interval was 19.0 ± 11.2 months (range 12–32 months). No significant differences were found among the patients concerning patient gender, BMI, habit of smoking, and whether or not the patient had diabetes or suffered from spondylolisthesis (*P* > 0.05) (Table 1). ICC of HU values between two independent researchers was 0.97. The average HU value of lumbar vertebra was 122.4 ± 32.8 HU in the screw loosening group and 142.4 ± 38.2 HU in the control group, and the difference was significant (*P* < 0.001).

The article "Computed Tomography-Based Prediction of Lumbar Pedicle Screw Loosening" was published in 2023. Journal: Biomed Res Int.

Among potential risk factors of screw loosening, the incidence of pseudoarthrosis and the difference between the HU values of the lumbar vertebrae were the most significant. Considering that pseudoarthrosis could be the result of screw loosening, and that pseudoarthrosis can only be found during follow-up after surgery, and the purpose of the current study is to find the predictive factors for screw loosening, here we carried out ROC curve analysis on the HU values of the lumbar vertebrae to assess their diagnostic value for screw loosening. ROC curve analysis revealed that the average HU value of L1-L5 has relatively larger area under the curve (AUC) of 0.689 (95% CI: 0.605-0.773) (Figure 2).

However, ROC curve analysis failed to provide a cut-off HU value with high sensitivity and specificity to predict the incidence of screw loosening. Although pseudoarthrosis may not be the cause of screw loosening, it is correlated with clinical symptoms and the necessity for a revision surgery. Therefore, we chose specific HU value regions and, respectively, calculated the incidence of screw loosening and pseudoarthrosis in those regions. With the sensitivity of 68% and specificity of 57%, a HU cut-off value of ≤124 HU was a plausible cut-off point to predict screw loosening.

## 4. Discussion

Pedicle screw loosening is one of the main complications associated with internal fixation procedure in spine surgeries. It is responsible for failure of bone fusion, consistent pain, and reduced mobility. In some severe cases, a revision surgery is needed to alleviate those symptoms caused by pedicle screw loosening [13]. In previous studies, screw loosening was found to be more prevalent among patients with low bone density. This was considered to be due to the weakened screw-bone integration [14]. In vitro studies showed that specimens with low bone quality require significantly lower pull-out strength than normal controls, which can be translated into higher probability of pedicle screw loosening [15, 16]. It has been extensively reported that bone quality, especially the quality of cancellous bone, is the main contributor for stability of pedicle screw [17–19]. Here, in our research, the incidence of screw loosening was 20.5%, which is in accordance with previous reports.

Cement augmentation amid to increase screw-bone integration was used for screw anchorage for more than two decades. Although this method could increase the pull-out forces by twice as much as standard options, it may cause some fatal complications such as pulmonary cement embolism. Therefore, it is only rational to apply this technique only when the patient is in under high risk of screw loosening and its complications. The goal of our current research was to find a high sensitivity predictive reference from conventional computed tomography scans for postoperative screw loosening, and to help with the preoperative planning for measures for screw augmentation without increasing the medical bills or radiation foe patients. The previous research has already shown the correlations between bone mineral density and the incidence of screw loosening and the correlation of HU values in opportunistic CT scans with the results of qCT and dual X-ray absorptiometry (DEXA) tests [20]. The mean HU value was significantly lower in the screw loosening group than in the nonscrew loosening group, indicating the potential of HU value in predicting the incidence of screw loosening.

The article "Computed Tomography-Based Prediction of Lumbar Pedicle Screw Loosening" was published in 2023. Journal: Biomed Res Int.

Although there are no widely accepted methods to evaluate screw stability, several authors chose more than 1 mm of clear zone around screw to use as a reference to diagnose screw loosening [21, 22]. Sanden et al. achieved 64% sensitivity and 100% specificity by using this criteria [23]. Here, we used the threshold of 1 mm as the diagnostic standard for screw loosening.

The ratio of screw loosening was reported to be between 0 and 54.7 percent [24–28]. However, there are no consistencies regarding the patient age, gender, bone quality, and the standard for the diagnoses of screw loosening. In our study, the ratio of screw loosening was the highest at one year after surgery but decreased significantly during follow-up, indicating higher fusion success and increased vertebral stability.

Different cut-off values of HU were proposed by various authors to predict a high likelihood of screw loosening. In the study of Bokov [29], when the CT value of L3 vertebra is less than 81 HU, screw loosening is highly likely to be present after lumbar spine surgeries. Bredow et al. [30] proposed a cut-off HU value of 120 HU as an independent risk factor for screw loosening. When reviewing 215 patients, we found that a cut-off L1-L5 average HU value of 124 HU in the instrumented lumbar vertebra can be used as a reference for the application of screw augmentation measures to prevent screw loosening.

Regions for HU measurement were chosen manually by two independent observers in our study. This could raise concerns over the repeatability of those results. However, high intraclass correlation coefficients (ICCs) regarding interobserver reliability indicate high repeatability of this method.

The article "Computed Tomography-Based Prediction of Lumbar Pedicle Screw Loosening" was published in 2023. Journal: Biomed Res Int.

Screw loosening is considered a negative influencing factor for successful bone fusion. However, loosened screws do not necessarily lead to spinal instability that requires revision surgery. In our study, while the ratio of successful bone fusion was significantly higher in nonscrew loosening group than in the screw loosening group, the number of patients who needed revision surgery is not significantly different between the two groups. A larger sample size maybe needed to further verify the reliability of those cut-off points. While the current consensus on the pullout strength of pedicle screws is that approximately 80% of the caudocephalad stiffness and 60% of the pullout strength of the pedicle screw depended on the pedicle rather than the vertebral body [31], and that the cancellous bone in the vertebral body accounts for approximately to 15-20% of the pull-out strength [32], the vertebral HU value reflects the bone mineral density of both pedicle and vertebral body; therefore, it can still be a useful indicator for the prediction of pedicle screw loosening. In the meanwhile, HU values of both the pedicle and the cancellous bone in the vertebral body could be used in combination to better predict the possibility of revision surgery due to screw loosening and the necessity for preventive measures such as pedicle screw augmentation.

## 5. Conclusion

A prospective CT scan HU value-based prediction can be used to decide whether or not to use screw augmentation methods. A cut-off L1-L5 average HU value of 124 HU can be used as independent risk factor for screw loosening in instrumented lumbar vertebra.

## Figures and Tables

**Figure 1:** A region of interest (ROI) within the cortex of the vertebra was determined on a horizontal plane at the level of pedicle, from which attenuation in HU was computationally generated.

**Figure 2:** ROC curve analysis on the predictive validity of HU value of different lumber vertebrae. ROC curve analysis revealed that the average HU value of L1-L5 has relatively larger area under the curve (AUC) of 0.689 (95% CI: 0.605-0.773).

**Table 1:** Demographic characteristics of the included patients in the two groups.

	Nonloosening	Loosening	*P*
Male/female	98/73	26/18	0.87
Age	57.4 ± 7.3	59.3 ± 7.9	0.15
Time of follow-up	18.7 ± 11.5	19.4 ± 10.8	0.71
BMI	25.4 ± 4.3	24.8 ± 4.6	0.42
Smoker	15	6	0.39
Diabetes	32	10	0.53
HU			
L1	149.6 ± 47.2	126.3 ± 40.8	<0.01
L2	143.7 ± 40.7	122.5 ± 35.7	<0.01
L3	134.6 ± 39.5	115.6 ± 36.2	<0.01
L4	133.2 ± 38.7	113.8 ± 34.8	<0.01
L5	150.8 ± 45.6	132.6 ± 39.7	<0.01
L1-5	142.4 ± 38.2	122.4 ± 32.8	<0.01

## Data Availability

All data generated or analyzed during the present study can be required from the corresponding author.

The article "Computed Tomography-Based Prediction of Lumbar Pedicle Screw Loosening" was published in 2023. Journal: Biomed Res Int.

## Abbreviations

HU: Hounsfield units
ANOVA: One-way analysis of variance
ROC: Receiver operating characteristic
AUC: Area under the curve
CT: Computed tomography
ROI: Region of interest
DEXA: Dual X-ray absorptiometry.
